The article "An Intervention Pattern of Family Parent-Child Physical Activity Based on a Smartphone App for Preschool Children during COVID-19" was published in 2022. Journal: Biomed Res Int.

# An Intervention Pattern of Family Parent-Child Physical Activity Based on a Smartphone App for Preschool Children during COVID-19

**DOI:** 10.1155/2022/2777079

**Published:** 2022-08-22

**Authors:** Xiaowei Han, Zhulin Tian, Meiling Zhao, Zhixiong Zhou

**Affiliations:** ^1^Faculty of Education, Beijing Normal University, Beijing 100875, China; ^2^Graduate School, Capital University of Physical Education and Sports, Beijing 100191, China; ^3^School of Physical Education and Coaching Science, Capital University of Physical Education and Sports, Beijing 100191, China

## Abstract

**Objective:**

Children's lifestyles, behaviors, and educational activities were affected by COVID-19. The preschool children struggled with the challenge of learning at home and avoiding a rapid decrease in physical activity (PA). This study tested the effectiveness of a family-based intervention that integrated the family and preschool based on a smartphone app to improve the moderate-to-vigorous PA (MVPA) and physical fitness of preschool children during COVID-19.

**Methods:**

This 8-week study was conducted using a quasiexperimental pre- and posttest design with a comparison group. A total of 66 pairs of preschool children (30 boys) and their parents and 44 preschool children (24 boys) and their parents composed the experimental group (EG) and the control group (CG), respectively. PA was measured using a GENEActiv waveform triaxial accelerometer. Children's physical fitness was assessed using a battery test from the Chinese National Measurement Standards on People's Physical Fitness for preschool children.

**Results:**

Preschool children and their parents in the EG participated in less sedentary (*p* < 0.01) and more light PA (*p* < 0.01) and MVPA (*p* < 0.01) compared with those in the CG at the late PA assessment. The EG significantly improved the mean performance of tennis ball throw (*p* < 0.05), balance beam walk (*p* < 0.01), and continuous jumping on both feet (*p* < 0.01) compared to the CG.

**Conclusions:**

The family parent-child PA intervention based on a smartphone app can effectively increase the MVPA of preschool children and their parents, reduce sedentary time, and improve preschool children's physical fitness. Overall, the family parent-child PA intervention model based on a smartphone app for preschool children designed in this study is feasible and effective.

## 1. Background

The coronavirus disease 2019 (COVID-19) pandemic is a public health emergency of international concern [1]. The World Health Organization (WHO) stressed and urged governments of all countries to remain vigilant and fully prepared to implement epidemic prevention measures [2]. COVID-19 has had a significant impact on people's lifestyles and school education activities, especially traditional school-based teaching activities. Schools have adopted a network-based teaching model to reduce the impact of the epidemic on children's learning in which children's learning places have been confined to home. As the teaching environment changes from school to family, guaranteeing the organized physical education curriculum and prescribed physical activity (PA) time is difficult. Consequently, the children's PA levels have significantly declined and not reached the international level [3]. During COVID-19, online physical education methods improved the physical fitness of adolescents [4]. In the last 10 years, several reviews reported that the efficacy of smartphone-based mHealth PA interventions could be considerably improved [5]. However, the studies targeting children or adolescents (age range: 5–19 years) were limited [5].

Higher levels of PA in preschoolers are positively associated with important benefits in physical [6–8], emotional, social, and cognitive domains [9–11] throughout life. Insufficient moderate-to-vigorous PA (MVPA) and prolonged sedentary activity and inactivity are some of the important problems to be solved urgently to promote children's physical health. Studies have pointed out that insufficient PA is an early risk factor for obesity in preschool children, and hence, the PA pattern of preschool children deserves attention [12, 13]. Currently, the epidemic of COVID-19 has brought challenges to the improvement in the PA levels of preschool children. During the epidemic, preschool children's lives and activities have been confined to home, and sports activities organized by teachers and with the participation of their peers are lacking. As a result, ensuring MVPA for preschool children is difficult [3]. The intervention method based on network application can break some obstacles existing in traditional intervention and has the advantages of not being limited by place and time, providing rich activities, and being easily accepted and used by parents and children [14]. A recent formative study has shown that parents are open to using digital applications to support preschool children's PA [15].

The main objective of the present study was to evaluate the effectiveness of a family parent-child PA intervention based on a smartphone app regarding the changes in the objective measurement of the PA of preschool children and their parents. We also investigated the effects of the intervention on the physical fitness of preschool children.

We hypothesized that, compared with children and parents in the control group (CG), the participants in the experimental group (EG) would show significantly greater increases in MVPA from baseline to postintervention time points, and the children in the EG would report higher levels of physical fitness.

## 2. Methods

### 2.1. Study Design and Sample

This was a pre- and posttest study with the CG using a quasiexperimental design. The study was conducted for 8 weeks from October 2020 to December 2020. For the sake of epidemic prevention and control in Beijing, the preschoolers did not go to kindergarten during this period and had activities at home. Two first-level public kindergartens were selected in the urban area of Beijing. The inclusion criteria were as follows: (1) availability of one parent and one child being in good health, (2) children's age between 3 and 5 years, and (3) the parent having a smartphone/iPad that could download and install apps and providing consent for themselves and their children to participate. The exclusion criteria were as follows: children who failed to wear the triaxial accelerometer to monitor PA in the experiment or who wore the triaxial accelerometer for fewer than three consecutive days.

Children aged 3–5 years were enrolled in three age-based grade levels. All children were invited to participate in the study. The parents were informed of the study via announcement posters at the beginning of the school year. All parents received consent letters and were asked to provide written consents for their children to participate in the study. No incentive was provided for participation in the study. The study protocol was approved by the ethics committee at the Capital University of Physical Education and Sports (code 2018072001) and registered in the Chinese Clinical Trial Registry (code ChiCTR1800017292).

A power calculation was conducted to estimate the required sample size. The calculations were conducted using G∗Power 3.1.9. Based on the mobile app on parent-child exercises [16], the intervention effect size of MVPA was estimated at *d* = 0.3. With a type *I* error probability of 0.05 and power of 0.8, the required sample size was calculated as 46. A minimum of 60 children were recruited to account for an estimated accelerometer noncompliance rate of 15% (i.e., cases with insufficient wear time) and a potential dropout rate of 20%. Based on the aforementioned inclusion and exclusion criteria, 110 pairs of eligible participants, including 66 pairs from the EG and 44 pairs from the CG, were enrolled in the final study analysis, meeting the requirements of statistical sample size.

### 2.2. Description of Intervention

#### 2.2.1. Theoretical Framework in the Intervention Design

The theoretical model used for the intervention was the Socioecological Model (SEM) [17]. This model recognized multiple levels of influence on health behavior and emphasized the complex interplay between individual, environmental, and policy contexts of healthy behavior. The PA habits of younger children were shaped by parents. Following the SEM, the study was designed to target combined parent-child PA.

#### 2.2.2. Intervention Design

The family-based PA intervention program for children and parents was designed by preschool exercise experts and early childhood educators based on SEM theory, physical and mental development characteristics of preschool children, and family environment characteristics. Based on the physical fitness and motor development approach, this intervention program comprised beneficial, enjoyable, and goal-directed family parent-child cooperative PAs, which included six kinds of PAs: running and climbing, jumping, throwing, balance, flexibility, and coordination. Considering the difference in professional sports equipment in the family environment and the cognitive ability of different parents, the intervention program designed in this study was simple and easy to understand. Also, the equipment required was simple and could be replaced by items at home. Parents could adjust it according to the actual situation. In the 8-week intervention cycle, the participants in the EG received 30 min of family PA intervention twice a week. The 8-week PA plan is shown in Table 1.

The study used the official account “YOUXUE UP” loaded on the WeChat app as an online intervention platform to implement family parent-child PA. This official account is an online teaching application platform developed by Beijing YOUXUE Partner Network Technology Co., Ltd., to provide schools, teachers, students, and parents with teacher-student interaction and home-school interaction services.  Figure 1 shows the framework of the app-based family parent-child PA intervention designed for this study.

Before starting the experimental intervention, 10 children and parents were invited to conduct a 1-week preexperiment. They were asked through a symposium about their experience in using the WeChat official account “YOUXUE UP” and their suggestions on the difficulty of designing the exercise content. The information obtained from the preexperiment was used to modify the process and practice content of the experimental intervention to improve the participation of the individuals. Before the formal experimental intervention, the researchers established a class through the WeChat official account “YOUXUE UP” and sent a class invitation link to the parents in the EG. After the parents registered successfully, they entered the class group. In addition, the researchers made short videos of each PA content and practiced precautions in preparing for the intervention. During the experimental intervention, the researchers sent preprepared practice tasks (short videos) to parents on time every Tuesday and Saturday (16:00–19:00 p.m.) through the WeChat official account of “YOUXUE UP.” The parents viewed through the official account, led their children to practice together at home according to the video requirements, and were required to record the practice process as a video and upload it. After the researchers received the feedback, they commented and scored in a timely manner. The parents could ask questions through the “mutual evaluation” of the official account. The researchers replied in time after receiving the feedback, and parents who had not uploaded the tasks received task reminders. According to the feedback, the researchers praised the children who completed all the tasks every week and provided small rewards as encouragement.  Figure 2 shows a screenshot of parent feedback on the completion of family parent-child PA.

#### 2.2.3. Control Conditions

During the experimental intervention period, the parents and children in the EG performed family parent-child PA based on the WeChat official account of “YOUXUE UP.” In the CG, the parents and children did not register the WeChat official account of “YOUXUE UP” to obtain the content of family parent-child PA. After the experiment, the parents in the CG register into the WeChat official account of “YOUXUE UP” free of charge to obtain resources for family parent-child PA.

### 2.3. Study Measurements

The main outcome variables of the study are shown in Table 2.

#### 2.3.1. Anthropometry

Height (cm) and weight (kg) were measured without shoes and with light, sports clothing with a stadiometer (SECA 213, Hamburg, Germany) and a balance scale (MIUI 2, Anhui, China), respectively. Body mass index (BMI) was calculated as weight in kilograms divided by the square of height in meters.

#### 2.3.2. Primary Outcomes

The PA of preschool children and their parents was measured using a GENEActiv waveform triaxial accelerometer (ActivInsights Ltd., Cambridge, UK). The parents of preschool children were informed about the precautions for wearing the GENEActiv accelerometer before testing to ensure that the accelerometer was properly worn. Preschoolers and their parents were required to wear the accelerometer on the wrist of the nondominant hand for seven consecutive days at two different test time points. The data for baseline PA were collected 1 week before the intervention (week 0), whereas the data for late PA were collected in weeks 6–7 of the intervention (week 6 or week 7). Due to the young age of preschool children, it was difficult to wear the accelerometer for a long time. If the valid data of the participant's accelerometer reached more than 3 days (including 1 day on weekends and 2 days during the week), it was included in the final data analysis. A total of 123 pairs of preschool children and their parents wore accelerometers, and 8 pairs of preschool children and their parents were excluded from incomplete accelerometer data records, resulting in 115 pairs of valid data. For each epoch (seconds), the motion data (activity counts) were added, recorded, processed, and analyzed. Cumulative activity counts were categorized by intensity into sedentary, light PA (LPA), and MVPA. The acquired data (.bin format) were processed by R software using R-Markdown provided by ActivInsights Ltd. For PA cut-points, the preschoolers used published cut-points [18], whereas the parents used R-Default cut-points in Markdown.

#### 2.3.3. Secondary Outcomes

A battery test from the Chinese National Measurement Standards on People's Physical Fitness for young children was used to assess children's physical fitness, which was defined as the body's ability to achieve optimal levels of physical performance in dealing with physiological stress to the body [19]. This normed assessment was validated in Chinese preschool-age children and used in the Chinese national fitness surveys [20]. The measurements included the standing long jump test for lower-body muscular strength, tennis ball throw test for upper-limb muscular strength, continuous jump on both feet test for coordination and lower-body muscular strength, 2 × 10 m SRT test for speed agility, sit-and-reach test for flexibility, and balance beam walk test for dynamic balance. The physical fitness indicators of children were tested 1 week before the intervention and 1 week after the intervention, and these tests were completed in kindergarten.

### 2.4. Statistical Analysis

SPSS 24.0 software (IBM Corporation, NY, USA) was used for statistical analysis of all data. The independent-sample *t*-test (height, weight, and BMI) and the chi-squared test (sex) were used to test for the differences in demographic variables. Then, 2 (group : EG and CG) × 2 (time : pre‐and posttest) repeated-measures analysis of variance was used to test the difference in the effect of experimental intervention. When the group×time interaction or the time and group main effects were significant, pairwise comparisons with statistical differences were further performed by simple-effects analysis. The partial *η*^2^ (*η*_*p*_^2^) was used as a measure of effect size and divided into small (0.01), medium (0.03), and large (0.14) effects according to Cohen's study [21]. A *p* value < 0.05 indicated a significant difference. All data were presented as the mean ± standard deviation (*M* ± SD).

## 3. Results

### 3.1. Characteristics of the Study Sample

In this study, 135 parents agreed to participate in the experiment, with a participation rate of 91.11%. A total of 110 pairs of participants participated in the pre- and posttests, and the dropout rate for the experiment was 10.57%. Further, 66 preschool children (age 4.16 ± 0.55 years, 45% boys) and their parents in the EG and 44 preschool children (age 4 ± 0.47 years, 55% boys) and their parents in the CG completed all the tests.  Figure 1 shows the participation process. The average weekly task completion feedback rate of the EG families was 65%. None of the participants experienced injuries related to the test or training content throughout the study period. This study analyzed the data of children (*N* = 110) who participated in the pre- and postexperiment tests. At baseline, no significant differences were found in demographic characteristics and primary and secondary outcome variables between the EG and CG (Table 3).  Figure 3 presents a flowchart of the participant selection process.

### 3.2. Intervention Effects on Primary Outcomes

Repeated-measures variance results showed that preschool children's sedentary (*F*(1, 105) = 37.59, *p* < 0.01, *η*_*p*_^2^ = 0.26), LPA (*F*(1, 105) = 22.37, *p* < 0.01, *η*_*p*_^2^ = 0.18), and MVPA (*F*(1, 105) = 347.86, *p* < 0.01, *η*_*p*_^2^ = 0.77) had significant interaction effects. A simple-effects analysis showed that the preschool children in the EG participated in less sedentary (*p* < 0.01) and more LPA (*p* < 0.01) and MVPA (*p* < 0.01) compared with those in the CG after the intervention. Compared with that at the baseline PA assessment, the preschool children in the EG participated in less sedentary (*p* < 0.01) and more LPA (*p* < 0.01) and MVPA (*p* < 0.01) at the late PA assessment, but no significant change was observed in the CG (*p* > 0.05) (Table 4).

Repeated-measures variance results showed that parents of preschool children with sedentary (*F*(1, 105) = 44.82, *p* < 0.01, *η*_*p*_^2^ = 0.3), LPA (*F*(1, 105) = 17.36, *p* < 0.01, *η*_*p*_^2^ = 0.14), and MVPA (*F*(1, 105) = 308.97, *p* < 0.01, *η*_*p*_^2^ = 0.75) had significant interaction effects. The simple-effects analysis showed that, compared with the CG, the parents of the preschool children in the EG participated in less sedentary (*p* < 0.01) and more LPA (*p* < 0.01) and MVPA (*p* < 0.01) compared with those in the CG at the late PA assessment. Compared with that at the baseline PA assessment, the parents of the preschool children in the EG participated in less sedentary (*p* < 0.01) and more LPA (*p* < 0.01) and MVPA (*p* < 0.01) at the late PA assessment. However, no significant change was noted in the CG (*p* > 0.05) (Table 4).

### 3.3. Intervention Effects on Secondary Outcomes

Repeated-measures variance results showed that preschool children's standing long jump (*F*(1, 105) = 17.98, *p* < 0.01, *η*_*p*_^2^ = 0.15), tennis ball throw (*F*(1, 105) = 8, *p* < 0.01, *η*_*p*_^2^ = 0.08), 2 × 10 m SRT (*F*(1, 105) = 14.93, *p* < 0.01, *η*_*p*_^2^ = 0.12), and balance beam walk (*F*(1, 105) = 19.05, *p* < 0.01, *η*_*p*_^2^ = 0.15) had significant interaction effects. The simple-effects analysis showed significantly greater improvements in the mean performances of tennis ball throw (*p* < 0.05) and balance beam walk (*p* < 0.01) in the EG after intervention, as compared to the CG. Regarding the mean within-group changes, both groups significantly increased the mean of standing long jump, tennis ball throw, 2 × 10 m SRT, and balance beam walk from pre- to posttests (*p* < 0.05). In addition, the results showed a significant group main effect of continuous jumping on both feet (*F*(1, 105) = 5.57, *p* < 0.05, *η*_*p*_^2^ = 0.05). The simple-effect analysis showed significantly greater improvements in the mean performances of continuous jumping on both feet in EG after intervention, as compared to the CG (*p* < 0.01). With respect to mean within-group changes, EG significantly increased the mean of continuous jumping on both feet from pre- to posttests (*p* < 0.01), but not in CG (*p* > 0.05). Besides that, no significant interaction and main effects were found for sit-and-reach (Table 5).

## 4. Discussion

This study explored the feasibility and effectiveness of an online platform-based PA intervention model for preschool children's families during the COVID-19 epidemic. In the case of school suspension during the epidemic period, the content of family sports activities suitable for the physical and mental development of preschool children was provided to parents to improve the level of MVPA and physical health of preschool children using the model based on the online platform. The main findings of this study were that the family PA intervention based on a smartphone app effectively reduced the sedentary behavior of preschool children and their parents, improved their LPA and MVPA, and effectively improved preschool children's physical fitness, such as muscle strength, coordination, speed-agility, and balance.

A recently published review analyzed nearly 6 years of research published on digital intervention strategies to improve PA in preschoolers. It found that implementing child-centered digital PA interventions in kindergartens significantly improved physical activity in preschoolers, but implementing digital PA interventions monitored only by parents was not effective in improving PA levels in preschoolers [22]. The main reason for this result was that the parents played only a supervisory role in the interventions included in the analysis and did not participate in the practice with their children through the same intervention. Another possible reason was the use of subjective measurement tools to measure PA, which might be missed by subjective assessments due to the typical short-term, discontinuous PA of preschoolers. Objective measures may be more conducive to obtaining accurate data on the PA of preschoolers. A previous review also indicated that an objective accelerometer should be used to assess the PA levels of preschool children during PA intervention [23]. In this study, the designed family PA intervention plan needed to be completed by parents and children together, and the designed activities were more interesting. The participation rate in the EG reached 94%, which was widely praised by parents and children. Studies have shown that positive emotions are more conducive to improving children's enthusiasm for participation, and the fun and pleasure obtained during sports could encourage preschool children to participate more actively in PA [24, 25]. Moreover, the study also used an objective measurement tool to measure the PA of the participants, ensuring the reliability of the result data, which was also an important reason for the significant effect of this study.

In addition, the findings of the present study showed that the family PA intervention based on a smartphone app effectively improved preschool children's performance on standing long jump, tennis ball throw, 2 × 10 m SRT, balance beam walk, and continuous jump on both feet but had no significant effect on sit-and-reach. At the same time, this study also discovered that the preschool children in the CG have achieved significant improvement in standing long jump, tennis ball throw, 2 × 10 m SRT, and balance beam walk from pre- to posttests. Previous studies showed that some physical fitness in the CG after the intervention also significantly improved [26, 27], indicating that the current routine PA implemented in kindergartens had a certain effect in terms of improving some physical fitness of preschool children. However, when it comes to changes in preschool children's physical fitness, it is critical to evaluate not only the statistically significant changes across time but also the practical implications for results. The results acquired in this study demonstrated that the performances of tennis ball throw, balance beam walk, and continuous jump on both feet of preschool children in the EG were significantly better than those in the CG (*p* < 0.05) after intervention. In addition, preschool children in the EG improved significantly more than those in the CG on standing long jump, tennis ball throw, continuous jump on both feet, 2 × 10 m SRT, and balance beam walk from pre- to posttests (Table 5). These findings were similar to previous results [20, 26, 28]. A recent meta-analysis confirmed that the PA interventions in preschool children produced positive changes in lower-body strength and speed-agility [28]. Macak et al. showed that the daily PA designed for preschool children effectively improved their upper- and lower-body strength [26]. Zhou et al. pointed out that the policy-driven, multiagent participation in PA intervention effectively improved preschool children's physical fitness such as muscle strength, agility, balance, and coordination [20]. In this study, the preschool children in the EG showed significant improvements in muscle strength, coordination, speed-agility, and balance, mainly because the designed family parent-child sports activities included strength, motor coordination, stability, locomotor, and object control (e.g., frog jump, hopscotch, stand on each leg, spider crawl, and overhand throw), which effectively stimulated the physical development of preschool children. However, it should be noted that this intervention did not improve flexibility in preschool children, which was similar to the findings of Macak et al. [26]. Studies showed that flexibility decreased with age, and this decline was caused not only by aging-related changes but also by a lack of training in this flexibility, which can be maintained or improved by training in specific ways [29, 30]. Therefore, this study did not report that the possible reason for the improvement in preschool children's flexibility was due to the inclusion of less relevant exercises while designing the activities, which also needs to be improved in future research.

## 5. Strengths and Limitations of the Study

This study had several strengths. First of all, in the case of epidemic prevention and kindergarten suspension, an online platform-based parent-child PA intervention model for families with preschool children was established. Also, the family parent-child PA exercises were provided to parents through a smartphone app, which effectively improved the level of MVPA and physical fitness of preschool children. In addition, the family PA intervention program designed in this study was interesting and interactive and was deeply liked by preschool children and their parents, which was important for discovering positive intervention effects. Finally, this study used a triaxial accelerometer for the objective measurement of PA, which guaranteed the objectivity and accuracy of the PA results [23].

There were several weaknesses in the study. First, there was no follow-up to examine if the changes in physical activity and physical fitness were sustainable beyond the 8-week intervention. Second, the study used a nonrandomized design, and the sample size was relatively small. Third, this family-based PA was delivered in an unstructured context and nonprofessional organization. Although the applied programs were well designed and properly controlled, parents would still have to be fenced off by the expertise of their application, because they lack professional knowledge and skills in physical education. This refers primarily to the organizational aspect of the activity but certainly also to the dynamic and kinematic structure of individual exercises. Namely, it is known that this is the period of children's growth which is specific for numerous morphofunctional changes. Certainly, each exercise would have to have a specific application in terms of starting position, amplitude of movement, pace of execution, dosage, etc. Moreover, it is known how many harmful effects the phones themselves and their use near the youngest can produce, but now, it is being promoted as a transmitter of certain physical activity programs, which could leave a psychological effect on children in terms of highlighting the smartphone as a necessary tool for many life activities.

Besides that, the generalizability of our findings is limited due to the fact that this study was delivered to Chinese city families. Therefore, future research should include families who live in the countryside or in a cross-cultural context. Meanwhile, future research and policymakers should also aim to strengthen specifically targeting parents and children who are inactive or are at risk of health issues.

## 6. Conclusions

In the case of epidemic prevention and control and kindergarten suspension, the family parent-child PA intervention model for preschool children based on a smartphone app can effectively increase the MVPA of preschool children and their parents, reduce their sedentary time, and improve preschool children's physical fitness, such as muscle strength, coordination, speed-agility, and balance. Overall, the family parent-child PA intervention model based on a smartphone app for preschool children designed in this study is feasible and effective.

## Figures and Tables

**Figure 1:** Framework of the family parent-child PA intervention based on a smartphone app.

**Figure 2:** Screenshot of parent feedback on the completion of family parent-child PA.

**Figure 3:** Flowchart of the participant selection process.

**Table 1:** PA intervention plan based on a smartphone app.

Week	Week 1	Week 2	Week 3	Week 4

Content	Bear crawl	Overhand throw	“S” crawl	Ant crawl race
	Obstacle courses	Catch with both hands	Lying leg raise	Seated knee tucks
	Shuttle run	Catch with a container	Jump over rope	Shuttle run
	Ski jump	Jump with a ball squeeze	Frog jump	Bunny hop
	Cross jump	Jump forward and backward	Jump lunges	Burpee
	High knees in place	Hopscotch	Cross jump	Multidirectional run
	Standing fly	Fun toy (signal)	Walk rope	Stand on each leg

Week	Week 5	Week 6	Week 7	Week 8

Content	Jump-crawl combination	Spider crawl	Overhand throw	Jump squat
	Side slide	Seated knee tucks	Relay race	Jump jacks
	Jump jacks	Log roll	Lateral high knee	Jump lunges
	Jump lateral	High five lunge jump	Burpee	High knees and clap
	Hop	Squat punch	Standing leg curl	Fun chair (signal)
	Catch the tail	Single leg squat	“S” backward run	Jump obstacle and throw
	Shoulder presses	Parent-child yoga	Standing trunk twist	Duck walk

**Table 2:** Description of study outcome measurement.

Measure(s)	Purpose	Instrumentation
PA	To measure the levels of PA for preschool children and their parents [18].	PA was measured using a GENEActiv waveform triaxial accelerometer (ActivInsights Ltd., Cambridge, UK).
Weight and height	To calculate BMI (weight in kg/height in m^2^) as a measure of anthropometrics.	Weight using a stadiometer (SECA 213, Hamburg, Germany); height using a balance scale (MIUI 2, Anhui, China).
Physical fitness	To measure the levels of physical fitness for preschool children [19].	Standing long jump test for lower-body muscular strength, tennis ball throw test for upper-limb muscular strength, continuous jump on both feet test for coordination and lower-body muscular strength, 2 × 10 m SRT test for speed agility, sit-and-reach test for flexibility, and balance beam walk test for dynamic balance.

Note: BMI: body mass index; PA: physical activity; SRT: shuttle run test.

**Table 3:** Baseline demographic characteristics of participants (*N* = 110).

Variables	EG (*n* = 66)	CG (*n* = 44)	*p*
Age (year)	4.16 ± 0.55	4.33 ± 0.43	0.118
Sex (male/female)^a^	30/36	24/20	0.350
Height (cm)	107.51 ± 4.35	106.33 ± 6.17	0.276
Weight (kg)	18.17 ± 1.63	18.22 ± 1.92	0.873
BMI (kg/m^2^)	15.72 ± 1.07	16.2 ± 2.16	0.174

Note: EG: experimental group; CG: control group; ^a^the difference between the two groups tested using the chi-squared test.

**Table 4:** Effects of the intervention on primary outcomes according to group (*N* = 110).

Variables	Baseline PA	Late PA	Mean difference [95% CI]^b^	*η*_*p*_^2^
Sedentary (min)^%^				
CG	146.89 (25.19)	143.91 (28.87)	-2.97 [-13.44 to 7.5]	0
EG	148.31 (25.61)	102.45 (25.04)	-45.85 [-54.65 to -37.24]^##^	0.51
Mean difference [95% CI]^a^	1.42 [-7.65 to 12.3]	-41.46 [-51.39 to -30.16]^∗∗^		
LPA (min)^%^				
CG	100.6 (30.9)	100.72 (25.06)	0.13 [-9.66 to 10.6]	0
EG	101.32 (29.53)	133.47 (30.48)	32.15 [23.69 to 40.15]^##^	0.36
Mean difference [95% CI]^a^	0.72 [-11.68 to 12.24]	32.74 [20.77 to 42.69]^∗∗^		
MVPA (min)^%^				
CG	7.87 (2.43)	8.32 (2.65)	0.46 [-0.86 to 1.75]	0
EG	7.63 (2.91)	24.06 (4.12)	16.43 [15.37 to 17.5]^##^	0.9
Mean difference [95% CI]^a^	-0.23 [-1.53 to 0.57]	15.74 [14.09 to 16.93]^∗∗^		
Sedentary (min)^%^				
CG	166.3 (18.58)	163.92 (19.6)	-2.38 [-12.4 to 8.16]	0
EG	163.66 (22.27)	116.89 (30.8)	-46.77 [-55.33 to -38.55]^##^	0.54
Mean difference [95% CI]^a^	-2.64 [-10.51 to 5.53]	-47.02 [-57.7 to -36.92]^∗∗^		
LPA (min)^&^				
CG	107.32 (22.73)	108.99 (23.1)	1.67 [-7.84 to 11.06]	0
EG	107.39 (23.28)	134.6 (25.82)	27.22 [19.54 to 34.97]^##^	0.32
Mean difference [95% CI]^a^	0.07 [-8.81 to 9.17]	25.61 [16.23 to 35.43]^∗∗^		
MVPA (min)^&^				
CG	4.77 (2.98)	5.72 (1.98)	0.95 [-0.33 to 2.2]	0.02
EG	5.15 (2.8)	20.51 (4.18)	15.37 [14.35 to 16.41]^##^	0.89
Mean difference [95% CI]^a^	0.37 [-0.77 to 1.45]	14.8 [13.45 to 16.12]^∗∗^		

Values are the observed mean (SD); all comparisons are adjusted for sex, age, and BMI. Note: CG: control group; EG: experimental group; PA: physical activity; LPA: light physical activity; MVPA: moderate-to-vigorous physical activity; ^%^preschool children; ^&^parent; ^a^mean between-group difference with 95% confidence interval based on estimated marginal means adjusted for sex, age, and BMI; ^b^mean within-group changes with 95% confidence interval based on estimated marginal means adjusted for sex, age, and BMI; *η*_*p*_^2^: partial eta squared; ^∗∗^*p* < 0.01 difference between CG and EG; ^##^*p* <0.01 difference between pre- and posttest.

**Table 5:** Effects of the intervention on secondary outcomes according to group (*N* = 110).

Variables	Pretest	Posttest	Mean difference [95% CI]^b^	*η*_*p*_^2^
Standing long jump (cm)				
CG	78.4 (13.9)	81.39 (12.86)	2.99 [0.53 to 5.62]^#^	0.05
EG	76.07 (14.32)	86.29 (10.14)	10.23 [8.1 to 12.24]^##^	0.47
Mean difference [95% CI]^a^	-2.33 [-1.14 to 9.26]	4.9 [-0.83 to 6.89]		
Tennis ball throw (m)				
CG	3.31 (1.13)	3.63 (1.15)	0.32 [0 to 0.65]^#^	0.04
EG	3.53 (1.28)	4.46 (1.43)	0.93 [0.66 to 1.19]^##^	0.32
Mean difference [95% CI]^a^	0.22 [-0.31 to 0.56]	0.83 [0.23 to 1.22]^∗∗^		
Continuous jump on both feet (s)^¥^				
CG	8.94 (3.18)	8.52 (2.99)	-0.41 [-1.11 to 0.31]	0.01
EG	7.79 (2.93)	6.74 (2.07)	-1.05 [-1.63 to-0.48]^##^	0.11
Mean difference [95% CI]^a^	1.15 [-2.32 to 0.02]	1.79 [-2.74 to-0.83]^∗∗^		
2 × 10 m SRT (s)^¥^				
CG	9.01 (1.53)	8.42 (1.26)	-0.58 [-0.82 to-0.19]^##^	0.09
EG	9.13 (1.72)	7.88 (0.98)	-1.25 [-1.56 to-1.05]^##^	0.49
Mean difference [95% CI]^a^	0.12 [-0.06 to 0.96]	-0.55 [-0.71 to 0.01]		
Sit-and-reach (cm)				
CG	11.36 (3.27)	10.92 (2.25)	-0.44 [-1.73 to 0.6]	0.01
EG	10.7 (4.42)	10.38 (3.8)	-0.32 [-1.19 to 0.71]	0
Mean difference [95% CI]^a^	-0.66 [-2.58 to 0.49]	-0.54 [-1.97 to 0.53]		
Balance beam walk (s)^¥^				
CG	13.83 (5.32)	11.68 (4.47)	-2.15 [-3.41 to-0.64]^##^	0.07
EG	15.01 (6.49)	9.11 (3.59)	-5.9 [-7.11 to-4.86]^##^	0.52
Mean difference [95% CI]^a^	1.18 [-0.36 to 4.03]	-2.56 [-3.54 to-0.71]^∗∗^		

Values are the observed mean (SD); all comparisons are adjusted for sex, age, and BMI. Note: CG: control group; EG: experimental group; ^¥^reverse scoring; ^a^mean between-groups difference with 95% confidence interval based on estimated marginal means adjusted for sex, age, and BMI; ^b^mean within-group changes with 95% confidence interval based on estimated marginal means adjusted for sex, age, and BMI; *η*_*p*_^2^: partial eta squared; ^∗^*p* < 0.05 difference between CG and IG; ^∗∗^*p* < 0.01 difference between CG and EG; ^#^*p* < 0.05 difference between pre- and posttest; ^##^*p* < 0.01 difference between pre- and posttest.

## Data Availability

The data used to support the findings of this study are included within the article. Further data or information is available from the corresponding author upon request.
